The article "Assessing Deep Learning Techniques for the Recognition of Tropical Disease in Images from Parasitological Exams" was retracted in 2023. Reasons: signs of a paper mill; suspected computer-generated content; unreliable results or conclusions; concerns about the data.

# Assessing Deep Learning Techniques for the Recognition of Tropical Disease in Images from Parasitological Exams

**DOI:** 10.1155/2022/2682287

**Published:** 2022-05-09

**Authors:** Ammar Akram Abdulrazzaq, Asaad T. Al-Douri, Abdulsattar Abdullah Hamad, Mustafa Musa Jaber, Zelalem Meraf

**Affiliations:** ^1^Department of Medical Laboratory Technologies, Al-Maarif University College, Ramadi, Iraq; ^2^Department of Dental Industry, College of Medical Technology, Al-Kitab University, Alton Kopru, Iraq; ^3^Department of Medical Laboratory Techniques, Dijlah University College, Baghdad 10021, Iraq; ^4^Department of Medical Laboratory Techniques, Al-Turath University College, Baghdad 10021, Iraq; ^5^Department of Medical Instruments Engineering Techniques, Al-Farahidi University, Baghdad 10021, Iraq; ^6^Department of Statistics, Injibara University, Injibara, Ethiopia

## Abstract

*Schistosoma mansoni* is one of the tropical diseases with the greatest epidemic reach in the world. One of the WHO guidelines is the prior and efficient diagnosis for mapping foci and applying the appropriate treatment of infected people. The current process for diagnosis still depends on an analysis of parasitological exams performed by a human being under a laboratory microscope. The area of pattern recognition in images presents itself as a promising alternative to support and automate image-based exams, and deep learning techniques have been successfully applied for this purpose. In order to automate this process, it is proposed in this work the application of deep learning methods for the detection of schistosomiasis eggs, and a comparison is made between two deep learning techniques, convolutional neural network (CNN) and structured pyramidal neural network (SPNN). The results obtained in a real database indicate that the techniques are effective in the recognition of schistosomiasis eggs, in which both obtained AUC (area under the curve) above 0.90, with the CNN showing superiority in this aspect. . However, the SPNN proved to be faster than the CNN.

## 1. Introduction

Schistosomiasis is one of the most endemic neglected tropical diseases in the world, according to the World Health Organization (WHO) [1]. Schistosomiasis is present in 76 countries across Africa, the Eastern Mediterranean, the Western Pacific, and the Americas. It is estimated that 200 million people are infected with the disease and 500 million people are exposed to risk areas [2]. In the Arabic region, the estimated number of individuals infected with schistosomiasis is 2.5 million people, but this number can reach 6.5 million due to lack of diagnosis or mapping of some endemic regions [3, 4]. There is still a lack of research that carries out mapping more endemic regions in the country. The most recent research was carried out using georeferenced data by field researchers to map the prevalence of schistosomiasis in the northeast region, more specifically in the coastal region of the state of Schaap et al. [4]. According to the London Declaration's definitions, the fight against schistosomiasis, according to the definitions of the London Declaration [5], involves the search for new techniques for diagnosis and mapping of the disease, which are easy to use, reliable, and low cost for patient monitoring and identification. With this, the aim is to observe the emerging behavior of this endemic. Computational techniques and new clinical analysis technologies are already widely used to support decision-making in the medical field and detect various diseases in medical image examinations. *Schistosoma mansoni* [6] is an infection caused by the schistosome (*Schistosoma mansoni*), a flatworm worm, a parasite of humans and some marsupial mammals, using the portal vein, responsible for conducting venous blood to the liver from various organs, for transmission of the adult worm. The disease diagnosis is performed by examining the parasite load collected from the feces. For the process of detecting and counting eggs in a sample, the Kato-Katz method [7] is used, which is currently considered the gold standard for egg counting and egg preparation of the blades. After this preparation, an analysis is performed using an optical microscope with a magnification of the objective lens 100 times. The count of schistosomiasis eggs present in the sample determines the parasite load and the degree of infection of the individual. The entire process is performed by a human manually. The lab technician looks for the following characteristics of the egg: lateral spine (spicule), irregular ellipsoidal shape with two enveloping membranes, and measuring about 115 mm in length and 65 mm in width.  Figure 1 shows an image of a parasitological examination with a *Schistosoma mansoni* egg detected, identified in the figure by a black rectangular border [8].

The article "Assessing Deep Learning Techniques for the Recognition of Tropical Disease in Images from Parasitological Exams" was retracted in 2023. Reasons: signs of a paper mill; suspected computer-generated content; unreliable results or conclusions; concerns about the data.

For health professionals working in nonendemic SM regions, the diagnosis of this entity can often not be remembered, and indeed, a thorough anamnesis, including information about the geographic history, exposure to potentially contaminated water or food, bathing in snail ponds, and trips to endemic areas. The occurrences of signs and symptoms of acute infection syndromes (especially cercarial dermatitis and Katayama fever), associated with physical examination findings, are essential elements for the presumptive diagnosis of SM. The naturalness of the patient is relevant for the appreciation of the picture. People from urban or unaffected areas, who have never had contact with *S. mansoni* and who, therefore, are devoid of immunity, often have acute episodes of the morbid condition with symptoms associated with an allergic condition. The acute forms of SM are closely related to ecological tourism and poor sanitation conditions. In contrast, individuals residing in endemic areas do not usually exhibit the manifestations of the acute phase [7, 8].

Indisputably, it is necessary to improve the techniques in use, tending to be aware and reduce the prevalence of parasitic loads. It is important to note that the easy identification of two eggs of *S. mansoni* makes false positive results unlikely. On the other hand, the relatively low sensitivity of direct demonstration techniques of evolutionary forms of parasites can be attenuated through refinements that increase the probability of being found in the material where they are still scarce. It is frequently necessary to use more than one coproscopic technique. Among the factors to ponder to be made to choose procedures for routine use is a trust-benefit relationship; it is opportunity to point out that some techniques become unnecessarily onerous.

The technique usually used in endemic control programs is that of Kato and Miura apud Komiya and Kobayashi, which modified by Katz et al. [9] went on to include the use of a sieve to remove macroscopic residues and a measuring plate to control the volume of the feces samples to be examined. Quantitative data are allowed to be obtained in terms of eggs per gram of feces (*opg*) or as well called the Kato-Katz method. It passed to be recommended by the World Health Organization and various authors, among them Mott, for employment in control programs for *Schistosoma mansoni*. Formerly, Abdullah Hamad et al. Molina, Coura and Conceição, and Dantas and Ferreira [7] have discussed the advantages and disadvantages of other techniques for coproscopic diagnosis of *S. mansoni*.

The deep learning techniques are generally implemented as artificial neural networks as opposed in their architecture by several hierarchical layers, being extensively explored recently, with significant success rates in the area of pattern recognition in images in the health area. Considering the recent success of these techniques, the present work proposes their application to implicitly extract the important characteristics of schistosomiasis eggs, aiming at their automatic diagnosis.

### 1.1. Theoretical Work

#### 1.1.1. Convolutional Neural Network (CNN)

The convolutional neural network (CNN) [10] is a feed forward network. They typically have the following layers in their architecture: convolutional layers, subsampling layers (or pooling), and dense layers (or fully connected), which can be arranged in different ways depending on the problem addressed.

The article "Assessing Deep Learning Techniques for the Recognition of Tropical Disease in Images from Parasitological Exams" was retracted in 2023. Reasons: signs of a paper mill; suspected computer-generated content; unreliable results or conclusions; concerns about the data.

The convolutional layers are responsible for spreading the data input and sharing the weights of the connections with the following layers. Each neuron is connected to a small set of the input vector, that is, to a small specific area, having similarity with the receptive fields of the human vision system. Different neurons in the convolutional layer account for different areas of the input data vector, overlapping to obtain a better representation of the input signal. The nodes of the convolutional layers are grouped in feature maps with the shared weight of the connections with the inputs acting as filters for each layer. This weight sharing significantly reduces the number of network parameters, increasing the efficiency and generalization capacity of the model. These convolutional layers have a nonlinear activation function to capture more complex properties of the input vector.

The subsampling layers, also known as pooling, segment the inputs of the previous layers into smaller groupings, reducing the sensitivity of the output to small variations and nuances of the data input. Generally, a maximum or average function is applied to the subsampling layer's input data to avoid the variations as mentioned earlier.

Finally, the dense layers, also known as fully connected, are applied as an activation layer for the classification process of the input set patterns.

Training a CNN is similar to other simpler techniques of the artificial neural network [11], where there is a minimization of the loss function using gradient descending and the backpropagation error. Developing a new CNN for a specific problem is not trivial, given the dependence of the configuration of each layer and the various parameters with the problem in question.

Some consolidated CNN architectures are already applied to image recognition problems, such as CifarNet, AlexNet, and GoogleLeNet. In this work, CifarNet was chosen, given the simplicity of the architecture, generating less effort to define the parameters.

#### 1.1.2. SPNN (Structured Pyramidal Neural Network)

The SPNN [12] is inspired by the pyramidal neural network (PyraNet) [13], which in turn was bioinspired by the concepts of receptive fields of human vision. The Pyrenees have two sets of layers: a 2D layer set and a 1D layer set. In the first set of 2D layers, each neuron is arranged in a matrix where each of the neurons is associated with a region of the predecessor layer, called the receptive field. In PyraNet, these receptive fields have a fixed size, and the 2D layers form a pyramid. The first layer of the 2D set, the base of the pyramid, is responsible for receiving the input image on the network. The other 2D layers are responsible for performing the implicit extraction of features from the input image and reducing the model's dimensionality. The set of 1D layers is placed on top of the pyramidal structure to perform the classification based on the features extracted by the predecessor layers. The SPNN is inspired by PyraNet and SOM networks (self-organized maps) and has a self-adaptive architecture, making the concept of a fixed receptive field more flexible. With these characteristics, the SPNN significantly reduces the number of parameters of the technique and the amount of resources needed to achieve a good detection rate. To construct the irregular receptive fields, the SPNN uses a probability map generated by the input images to determine the point cloud in the receptive fields. For constructing the regions of interest of the receptive field, the SPNN uses Delaunay triangulation [9]. The clustering algorithm K-means groups the points of interest from these regions, minimizing the number of neurons in the layers ahead. This process is repeated for the following layers until the last layer uses only one neuron. With this simpler architecture, the SPNN achieved promising results in previous works [14] when compared to more computationally expensive techniques, such as the CNN and SVM (support vector machine). SPNN training follows the same training model as other artificial neural networks, as presented for CNNs.

The article "Assessing Deep Learning Techniques for the Recognition of Tropical Disease in Images from Parasitological Exams" was retracted in 2023. Reasons: signs of a paper mill; suspected computer-generated content; unreliable results or conclusions; concerns about the data.

## 2. Methodology

The purpose of this work is to adapt two deep learning models, CNN and SPNN, for application in the detection of *Schistosoma mansoni* eggs on the basis of real images. In previous works [14, 15], other classic techniques such as Haar-like and AdaBoost were applied in the detection of schistosomiasis eggs. An accuracy of approximately 80% was obtained; this value was used as a reference for the tests performed in this work and the methodology for acquiring and balancing the image base used in the validation of the model. This section presents the experimental arrangement, the preprocessing image methodology, the description of the image base used, and a preliminary study of the influence of parameters on the SPNN performance.

### 2.1. Experimental Arrangement

For this comparative analysis, thirty simulations were performed for each proposed technique, in addition to a convergence study to determine the number of times needed in each case. CifarNet was the convolutional neural network architecture selected and implemented for the CNN experiments, as it applies to problems involving classification with few classes and low-resolution images. Compared to other techniques, such as AlexNet and GoogleLeNet, it has lower complexity and better performance for the case type in question.

The article "Assessing Deep Learning Techniques for the Recognition of Tropical Disease in Images from Parasitological Exams" was retracted in 2023. Reasons: signs of a paper mill; suspected computer-generated content; unreliable results or conclusions; concerns about the data.

CifarNet parameters followed their canonical definitions. Three convolutional layers, 03 (three) subsampling layers, and 01 (one) dense layer were defined, with the ReLU (rectified linear unit) being used as an activation function in the convolutional layers and the logistic sigmoid in the dense layer. CifarNet was implemented using the Keras library [16] with backend support for TensorFlow [14]. The SPNN has significant results in detecting patterns in images and a similar accuracy compared to more consolidated techniques such as the CNN and SVM, as proposed by Chaganti et al. [17]. Because it has few network configuration parameters and has been evaluated in previous works with different configurations on different bases, it was decided to evaluate the impact and influence of each parameter on the image base of schistosomiasis before defining the best architecture. To analyze the best configuration of the SPNN to be parameterized, the number of points to determine the point cloud and the number of neurons in the first pyramidal layer were evaluated. Due to the SPNN training time being significantly shorter when compared to the CNN, a committee architecture of SPNNs was also tested, with 05 (five) independently trained networks and decision using average as reference.

All tests were performed on an instance of EC2 (Elastic Cloud Computing) of AWS (Amazon Web Services) with an Octacore Intel Xeon E-2676 2.4 GHz server, with 16 (sixteen) GB of RAM and 01 (a) 80 GB SSD disk. The implementations of all models were developed implementing multithreaded support aiming at parallelism in the cores of the server's processor.

The performances of the tested configurations are presented using the ROC (receiver operating characteristic) curve that relates the rate of true positives to the rate of false positives. The accuracy of the ROC curve is determined by its AUC (area under the curve). For this database, the true positive rate represents the amount of schistosomiasis eggs detected over the total positive images in the database. As well as the false positive rate represents the number of artifacts incorrectly detected and given as positive, divided by the amount of negative images in the base.

### 2.2. Data Preparation and Image Base Description

Before the execution of the present work, there was no public schistosomiasis image bank available in the literature for evaluation. In the work developed by Ivašić-Kos et al. [18], the schisto system was built, a software for image acquisition of schistosomiasis eggs in laboratory slides. In cooperation with the author of the schisto system, the pick cells system was developed, as an evolution of the previous research work. This platform is capable of performing the detection of parasites in image exams, in addition to segmenting objects of interest in the images obtained. Pick cells allow you to create new image banks from the exams performed.

The article "Assessing Deep Learning Techniques for the Recognition of Tropical Disease in Images from Parasitological Exams" was retracted in 2023. Reasons: signs of a paper mill; suspected computer-generated content; unreliable results or conclusions; concerns about the data.

As shown in Figure 2, the system selects the object of interest through a bounding box, and after validating the diagnosis in the system, an image is generated. with the coordinates of the object's location linked to a log file, responsible for storing this information. Using these images and the log file containing the object's position information, a Python script was developed to segment the images into two groups: positive and negative. The positive images contemplate the schistosomiasis eggs and the negative images contemplate the background images and contain other artifacts of the original image. The construction of the image bank for the experiments consisted of these segmented images. Three hundred thirteen positive images (images that include one or more schistosomiasis eggs) and 1048 negative images were extracted from the pick cells system, with the original resolution of 320 by 240 pixels. After this extraction, the object segmentation technique was applied, generating a base of positive objects of 15754 images. The negative image base was also balanced, containing 15754 images. A 28 × 28 resolution was adopted for all objects in the base, in addition to converting all images to grayscale. For cross-validation, the k-fold technique was applied to validate the generalization of the applied models, dividing it into two sets: training and testing. The training set is composed of 11029 positive images and 11029 negative images. The test set included 4725 positive and 4725 negative images.

### 2.3. Influence of SPNN Parameters

Before the beginning of the experiments, the influence of the SPNN parameters was evaluated to determine which configuration would be compared to the CifarNet (CNN) technique. Some configurations of neurons in the first pyramidal layer (N1) and the number of initial points of the Point Cloud (NP) were empirically defined. The number of neurons was varied from 03 to 40 and the point cloud was varied from 60 to 140, as shown in Figure 3. The configuration with 03 neurons in the first pyramidal layer and with 60 points in the point cloud obtained the best result. Wilcox statistical tests were performed with *p*=0.05, for the configurations with 60 points in the point cloud. There was no statistical significance in the comparison. Due to this, all SPNN analyses adopted the configuration with 03 neurons in the first pyramidal layer and 60 points for the point cloud, reducing the complexity and computational cost of the implementation.

The article "Assessing Deep Learning Techniques for the Recognition of Tropical Disease in Images from Parasitological Exams" was retracted in 2023. Reasons: signs of a paper mill; suspected computer-generated content; unreliable results or conclusions; concerns about the data.

## 3. Results and Methods

For each proposed model, a convergence study was performed as a function of the number of iterations. The models were run with 50, 100, 150, and 200 iterations. CifarNet converged quickly, and the results are similar for all proposed iterations. Despite having presented an average AUC of 0.965 with 150 iterations, the model found greater stability when executed with 200 iterations and an average AUC of 0.955, as shown in Figure 4.

It is important to note that even with 200 iterations, the model presented outliers, indicating instability of the technique when applied to the image base of the experiment. The SPNN stabilized after 100 iterations with an average AUC of 0.911.

Even so, it obtained an average AUC of 0.913 with 200 iterations, as shown in Figure 5. It is important to highlight the stability of this model after it reaches convergence.

The average values found by the models as a function of the number of iterations are shown in Figure 5.

After performing the 30 simulations, with 200 iterations for each simulation, the CNN obtained an average AUC of 0.955, while the SPNN obtained an AUC *m* average of 0.913. Due to the significantly shorter training and evaluation time of the SPNN when compared to that of the CNN, a configuration composed of a committee of 5 empirically defined SPNNs was also tested to validate if there would be again at AUC. The determination of accuracy in the SPNNs committee was determined by means. As shown in Figure 3, this gain was verified and the SPNNs committee obtained an average AUC of 0.942.  Figure 6 shows the boxplot of the AUCs obtained for the SPNN, 5 SPNNs, and CNN committee. It is possible to verify that despite a higher average value of AUC, the CNN presents a greater amount of outliers when compared to the SPNN and the committee of SPNNs. The SPNN's committee showed greater stability when compared to the CNN.

### 3.1. CNN (CifarNet) and SPNN's Committee

Figure 3 shows the training time for the deep learning models covered, SPNN, committee with 5 SPNNs, and CNN, considering 30 simulations. It can be seen that the SPNN and the committee of 5 SPNNs are 20 times and 2.53 times faster than the CNN, respectively.

## 4. Conclusions and Future Work

Some contributions of this work regarding the applied deep learning techniques can be highlighted. Both the CNN and SPNN presented results with greater accuracy than the current reference technique applied to the diagnosis of schistosomiasis.

The article "Assessing Deep Learning Techniques for the Recognition of Tropical Disease in Images from Parasitological Exams" was retracted in 2023. Reasons: signs of a paper mill; suspected computer-generated content; unreliable results or conclusions; concerns about the data.

The CNN model analyzed, CifarNet, widely used in the literature in applications of pattern recognition in images, obtained a relevant accuracy regarding the detection of eggs in the images of the experiment. Despite the instability, the speed of convergence was the positive factor regarding the application of this technique in the experiments.

The SPNN, a technique applicable to the detection of patterns in images, showed promising results and obtained greater stability compared to the CNN. As it obtained better performance in training and validation compared to the CNN, the implementation of an experiment contemplating a committee with 5 SPNNs guaranteed an increase in accuracy and greater stability, even when compared with the configuration of a simple SPNN and with CNN.

Due to the simplicity of the technique and the lower computational cost, SPNNs, when used in a committee, present relevant characteristics embedded in some low-cost technology. With this, the technology can be used at scale to detect schistosomiasis, which would meet one of the requirements of the millennium goals regarding the eradication of this disease.

The proposals for future works are to deepen the study of the two techniques regarding other parameters or definitions of network architecture and to observe if there is a possibility of improving the accuracy itself. There is also a need to compare the techniques evaluated with other nondeep models, such as SVM, to carry out more comprehensive studies of this application. It is still necessary to study the performance and suitability of these techniques for implementation in embedded systems, aiming to develop some support tools for improvements in the clinical analysis process. In the detection of schistosomiasis, another possibility is to expand the proposed techniques for detecting other geohelminthoses and neglected diseases, validating the generalization of the models used.

## Figures and Tables

**Figure 1:** Illustration of the *Schistosoma mansoni* egg.

**Figure 2:** Pick cells system segmenting images of schistosomiasis eggs.

**Figure 3:** Comparison of performance in terms of AUC for the deep learning models addressed: SPNN, committee with 5 SPNNs, and CNN.

**Figure 4:** Influence of the number of neurons in the first pyramidal layer (N1) and in the point cloud (NP) of the SPNN.

**Figure 5:** (a) CNN convergence analysis (CifarNet). (b) SPNN convergence analysis. (c) Comparison of the SPNN convergence with the CNN (CifarNet).

**Figure 6:** Training time of the deep learning models addressed: SPNN, committee with 5 SPNNs, and CNN, considering 30 simulations.

The article "Assessing Deep Learning Techniques for the Recognition of Tropical Disease in Images from Parasitological Exams" was retracted in 2023. Reasons: signs of a paper mill; suspected computer-generated content; unreliable results or conclusions; concerns about the data.

## Data Availability

The data used to support the findings of this study are included within the article.
